# Dendritic Cell Vaccine Loaded with MG-7 Antigen Induces Cytotoxic T Lymphocyte Responses against Gastric Cancer

**DOI:** 10.1155/2022/1964081

**Published:** 2022-04-18

**Authors:** Bohui Zhu, Yiyuan Sun, Xiaoqing Wei, Huibin Zhou, Jingchen Cao, Chenwei Li, Ning Wu

**Affiliations:** ^1^Department of Oncology, Shanghai Pudong New Area Gongli Hospital, Shanghai 200127, China; ^2^Shanghai Sunstem Biotechnology Co., Ltd., Pudong, Shanghai 200127, China

## Abstract

Dendritic cells (DCs) are antigen-presenting cells that can activate T cells and initiate a primary immune response. Personalized DC vaccines have demonstrated a modest antitumor potential in some clinical pilot studies. However, those vaccines are difficult to manufacture and have a limited antitumor response. In this study, a lentiviral vector-programmed DC vaccine with high antitumor responses is developed. By transfecting with a lentiviral vector, the DC vaccine is loaded with MG-7 antigen (MG-7Ag). Three representative gastric cancer cell lines, such as KATO-3, MKN45, and SNU16, are used to estimate the in vitro cytotoxic effect of the MG-7Ag DC vaccine. Furthermore, we examine the in vivo antitumor efficacy of specific cytotoxic T lymphocytes (CTLs) induced by the MG-7Ag DC vaccine in patient-derived xenograft (PDX) mice models. The current data demonstrate that the MG-7Ag DC vaccine induced a potent CTL activity. Those CTLs have a significant cytotoxic effect on both KATO-3 and MKN45 with high level of MG-7 expression. In addition, MG-7Ag DC vaccine-mediated CTLs significantly inhibit the growth of tumor xenografts in nude mice. The MG-7Ag DC vaccine activate the cytotoxic effect of lymphocytes and can be employed as a vaccine in gastric cancer immunotherapy.

## 1. Introduction

As the fifth frequently diagnosed cancer, gastric cancer causes approximately 783000 deaths and more than 1000000 new cases in 2018, which is regarded as the third most common cause of cancer-related deaths throughout the world [1]. The incidence rate of gastric cancer is higher in Eastern Asia (Japan, China, and the Republic of Korea) than in other regions [2]. In China, about 679100 newly diagnosed cases and 498000 deaths from gastric cancer were estimated in 2015 [3], and this type of cancer is the second leading cause of cancer-related deaths in China [4]. Traditional treatment, including surgical resection, radiation therapy, and chemotherapy, has not increased the 5-year overall survival rate for gastric cancer patients [5]. Thus, it is imperative to develop new therapeutic alternatives. Immunotherapy is regarded as a promising strategy that complements the current cancer therapies. Some malignant tumors, such as nonsmall cell lung cancer and melanoma, appear to benefit from immunotherapy [6], and a cancer vaccine is a critical part of this therapy. Dendritic cells (DCs) activate T cells to become cytotoxic T lymphocytes (CTLs) and initiate a primary immune response [7]. The current DC vaccines constitute a tumor therapy strategy that activates the immune system, and promising results have been obtained [8–10], which are safe and effective [11].

The current substances for antigen loading in the DC vaccine comprise DNA, synthetic peptides, whole tumor RNA, and tumor cell lysates [12]. Among these, the antigen-loading strategy using whole tumor cells is commonly used; however, DCs loaded with such lysates have stimulated only limited responses in a wide range of clinical trials, and these DC vaccines are difficult to manufacture and industrialize. Some studies have demonstrated lentiviral vector-programmed DCs, and this new method has a high potency and can be automatized [13]. MG-7 antigen (MG-7Ag) is a specific antigen of gastric cancer screened by the corresponding antibody, which is highly expressed in gastric cancer tissues but not in normal tissues [14]. MG-7Ag is a monoclonal antibody against gastric cancer prepared by immunizing mice with gastric cancer cell line MKN-46-9 as immunogen. MG-7Ag recognized by MG-7Ag is a newly discovered gastric cancer-related antigen. MG-7Ag is a neutral glycolipid. The epitope is located on the sugar chain. It is a glycoprotein antigen. It has the characteristics of secretory antigen, that is, it is synthesized in cells and then secreted outside cells. MG-7Ag can be roughly divided into four types in cells: cytoplasmic type, membrane type, extracellular type, and mixed type. The expression of MG-7Ag in gastric cancer has a relative tendency of histological type. The changes of morphology, biochemistry, and antigenicity of gastric mucosal epithelial cells in the process of carcinogenesis are related to gene damage and control imbalance [15]. Due to different genetic changes, the antigen expression order and tissue type of different types of gastric cancer are also different. Importantly, the prognosis for those with MG-7Ag-positive gastric cancer is worse than for those with MG-7Ag-negative gastric cancer.

## 2. Related Work

Gastric cancer is the fifth most commonly diagnosed cancer and the third most common cause of cancer-related deaths worldwide [16]. The incidence rates of gastric cancer are high in East Asian countries, such as Japan, China, and Korea. With nearly 500000 deaths annually, gastric cancer is the second leading cause of death in China.

Traditional surgery, radiotherapy, and chemotherapy cannot resolve the metastasis and recurrence of these tumors; therefore, new techniques are needed to break through the bottleneck of tumor therapy. Because it is safe and clinically effective, tumor autologous immune cell therapy is the best systemic therapy for tumor patients [17]. After development for more than 50 years, immune cell therapy has become the fourth most used method in tumor treatment after secondary surgery, radiotherapy, and chemotherapy. A cancer vaccine is a major part of immunotherapy. It is used to activate the immune system and induce a specific immune response against tumor cells. The DC vaccine is a cancer vaccine and a robust antigen-presenting cell because it can stimulate the proliferation of T cells. It is the initiator of the body's immune response and a natural “immune adjuvant” [18]. DC-based cancer vaccines aim to stimulate anticancer immunity by harnessing the capacity of DCs to activate specific T cells to become CTLs. In 2010, sipuleucel-T (Provenge) was approved by the United States Federal Drug Administration (FDA) to treat advanced prostate cancer. This was the first and only FDA-approved DC cancer vaccine [19, 20]. In recent years, some achievements have been made in the study of a gastric cancer DC vaccine [21–23].

MG-7Ag is a sensitive and specific antigen for gastric cancer screened by the corresponding antibody. The detection of gastric mucosal tissue by immunohistochemistry shows that MG-7Ag is highly expressed in superficial gastritis, atrophic gastritis, intestinal metaplasia, atypical hyperplasia, and gastric cancer [15], and the positive rate in gastric cancer is 82.8% [24]. Han et al. [25] used phage display library technology to successfully screen the mimotope peptide of gastric cancer MG-7Ag. In vitro studies have confirmed that the mimotope peptide mimics the original antigen and induces immunity against gastric cancer; the oral DNA vaccine for gastric cancer MG-7Ag-mimic epitope was developed using attenuated *Salmonella typhimurium*, and the immune efficacy of the vaccine was observed after immunizing mice [26]. Tumor antigens are critical in the preparation of vaccines, but the presentation of antigens is also essential [27]. We used lentivirus as a delivery vehicle because this vector has many advantages. For example, the lentiviral vector can transfect cells that divide slowly and at the end of the division, such as DCs. In addition, it can transfer gene fragments for target gene expression, making it difficult to induce an immune response.

In this study, we developed a DC vaccine loaded with MG-7Ag by transfecting with lentiviral vector. At the cellular level, the DC vaccine was used to stimulate T cells to form CTLs, and the cytotoxic effects of CTLs were evaluated on three gastric cancer cell lines. The results showed that the MG-7Ag DC vaccine-mediated CTL had a satisfactory cytotoxic effect on both KATO-3 and MKN45 cells, in which MG-7 was highly expressed. The cell killing indicated that specific monoclonal antigen DC vaccine-mediated CTL had a better killing effect on high-expression cells. Similarly, the DC vaccine loaded with MG-7Ag at the animal level also exhibited a tumor-inhibiting effect. Compared to that in the control and NC groups, the cytotoxic effect of the MG-7Ag DC vaccine-mediated CTL was the best. The MG-7Ag DC vaccine-mediated CTLs significantly inhibited tumor growth. We determined the cytotoxic effect of the MG-7Ag DC vaccine on gastric cancer. Thus, the DC cell vaccine was injected intravenously into the subjects, and the clinical effect was determined by observing and detecting the size of solid tumors and the specific sensitive antigen content of gastric cancer in blood. Finally, we obtained an effective DC cell vaccine for gastric cancer treatment.

## 3. Proposed Methods

### 3.1. Cell Lines and Animals

KATO-3, MKN45, and SNU16 cell lines were purchased from Shanghai Enzyme Research Biotechnology Co., Ltd., China. KATO-3 cells were cultured in Dulbecco's modified Eagle's medium (DMEM, Life Technologies, San Diego, CA, USA) containing 20% fetal bovine serum (FBS, Life Technologies) and 1% penicillin-streptomycin (Sigma-Aldrich, St. Louis, MO, USA). MKN45 and SNU16 cells were cultured in RPMI 1640 medium (Life Technologies) containing 10% FBS and 1% penicillin-streptomycin. Male NOD/SCID mice, 8 weeks old, were purchased from Shanghai SLAC Laboratory Animal Co., Ltd. All animal studies were conducted at the Shanghai Laboratory Animal Center, Shanghai, China.

### 3.2. Real-Time Quantitative Polymerase Chain Reaction

The RNA extraction kit (TaKaRa, Beijing, China) was used to extract total cell RNA, and a reverse transcription kit (TaKaRa) was used to reverse transcribe the total RNA into cDNA. The cDNA concentration was measured on a microplate reader. The forward and reverse primer sequences were as follows: 5′-CATACAAAAGGAGGAG GAAGTAAG-3′, 5′-CAGGTGGCTGTGGGGTTTA-3′. Glyceraldehyde 3-phosphate dehydrogenase served as an internal control.

### 3.3. Patient-Derived Xenograft Models

NOD/SCID mice were anesthetized intraperitoneally with 50 mg/kg pentobarbital and placed in a stereotactic frame. Gastric cancer tumor tissue was removed from liquid nitrogen to thaw and sliced into 4 mm^3^ pieces to subcutaneously inoculate into the mice. The mice were observed and weighed every 2 d.

### 3.4. Construction of MG-7Ag Lentiviral Vector

A synthetic fragment of MG-7Ag and carrier shRNA were digested with AscI and XbaI (TaKaRa) and analyzed by agarose gel electrophoresis. The target gene fragments and shRNA (+) fragments were excised from the gel. The MG-7Ag fragment was ligated to the vector overnight using T4 DNA ligase at 16°C. The ligation product was transformed into *Escherichia coli* DH5, and positive clones were screened on ampicillin-resistance plates and validated by polymerase chain reaction (PCR) (5′-CGCAAATGGGCGGTAGGCGTG-3′, 5′-CATAGCGTAAAAGG AGCAACA-3′) and sequencing.

### 3.5. Lentiviral Packaging

HEK-293FT cells were cultured in a Petri dish 10 cm in diameter. The serum-free medium was replaced 2 h before transfection. The DNA (containing expression plasmids pLVX-MG-7 and packaging plasmid pLP1, pLP2, and pLP/VSVG) was transfected into the cells using calcium phosphate [16]. The mixture was incubated under 5% CO_2_ at 37°C for 6 h, after which the medium was replaced and incubation continued for 2-3 d. The supernatant was collected by cell centrifugation at 4000 ×g at 4°C for 10 min, filtered through a 0.45 m filter, and centrifuged again using a Beckman ultracentrifuge (Beckman Coulter, Brea, CA, USA) at 4°C and 25000 rpm for 2 h. The supernatant was discarded, and the pellet was resuspended in the virus preservation solution and centrifuged at 10000 rpm for 5 min, after which the physical status and sterility were assessed, and the viral titer of the lentivirus was calculated using the following formula: virus titer = number of fluorescent cells/amount of virus stock [17].

### 3.6. Preparation of DC Vaccines

Peripheral blood mononuclear cells (PBMCs) were isolated from patients' peripheral blood using Ficoll-Hypaque (Solarbio, Beijing, China) and cultured in RPMI 1640 containing 5% autologous plasma, 10 ng/mL hGM-CSF (Miltenyi Biotec, Bergisch Gladbach, Germany), and 10 ng/mL hIL-4 (Miltenyi Biotec). The immature DCs were infected with lentivirus on day 5, and polybrene (transfection enhancer) was added. Fresh medium was replaced after 24 h of transfection, and poly I : C was added on day 6 to promote the expression of endogenous genes. The mature DCs were then collected on day 7. The maturation status of DCs was observed through a microscope (Leica Microsystems Inc., Wetzlar, Germany). The expression of CD80, CD83, CD86, and human leukocyte antigen (locus) DR (HLA-DR) in DCs were measured by flow cytometry (Beckman Coulter). To assess DC maturation, flow cytometry and enzyme-linked immunosorbent assay (ELISA) were used to detect secreted cytokines. MG-7Ag expression in DCs was detected by quantitative PCR (qPCR) and gel electrophoresis.

### 3.7. Study Design

T cells were cocultured with DCs (at a responder-to-stimulator ratio of 10 : 1) in the presence of 0.2 ng/mL hIL-2 (Miltenyi Biotec) at 37°C for 48 h. Then, CTLs were harvested and used as effector cells to detect CTL cytotoxicity; gastric cancer cells KATO-3 and MKN45 were selected as target cells, and CCK-8 (Shanghai Yeasen Biological Technology Co., Ltd, Shanghai, China) assay was used to determine the inhibition of CTLs on two gastric cancer cell lines in vitro.

To further verify the cytotoxic effect of DC vaccine-mediated CTL, a PDX mouse model was established and divided into the following three groups: control, negative control (NC), and MG-7Ag (*n* = 6 mice/group). The mice in MG-7Ag and NC groups were infused with normal saline solution, and those in the control group were infused with simple normal saline with CTL through a tail vein once a day for 3 consecutive days. The diameters of the tumor were measured using Vernier calipers, the weight of mice was measured, and the changes in tumor growth and mouse weight were plotted. Besides, the changes in the tumor were observed for 22 d.

### 3.8. Statistical Analyses

SPSS 16.0 (SPSS Inc., Chicago, USA) was used for biostatistical analyses, and the baseline description analysis was conducted. The Kaplan–Meier method was used to analyze survival, and the differences among the groups were compared using the log-rank test. *P* < 0.05 indicated statistical significance.

## 4. Results Analysis

### 4.1. Screened Cell Lines That Express MG-7Ag Target Antigen

To reflect how the MG-7Ag DC vaccine inhibited cancer growth, we measured the content of MG-7Ag in the gastric cancer cell lines and found that MKN45 and KATO-3 had high expressions of MG-7Ag, while cell lines NUGC-4, NCI-N87, SNU16, and SNU-5 had low expressions, as shown in Figure 1. Total RNA is isolated from LoVo, NUGC-4, NCI-N87, SNU16, SNU-5, MKN45, and KATO-3 cell lines, reverse transcribed to cDNA, and amplified by qPCR to evaluate MG-7Ag expression. The LoVo (intestinal cancer) cell line is used as a control.

### 4.2. DCs Express High Levels of Surface Markers

To cultivate high-quality DCs, we optimized the DC culture conditions. Mature DCs were characterized by high expression of MHC I, MHC II, CD80, CD83, CD86, and other costimulatory molecules, which process and present antigens for T cell recognition. Naive T cells could be activated only by mature DCs to convert them into CTLs that exert an antiinfective effect. Next, we estimate the surface markers CD80, CD83, CD86, and HLA-DR of DCs and found that after adopting our DC culture program, the expression levels of the DC surface markers markedly improved, as shown in Figure 2. These results further indicated that the DCs cultivated in the present study could induce CTL responses and regulate immune responses. The mature DCs were collected, washed, and resuspended in PBS. The experimental group containing 10 L of HLA-DR, CD80, CD83, and CD86 flow cytometry antibodies and the blank control group were incubated in the dark at 4°C for 30 min for testing.

### 4.3. DC Vaccine Can Express MG-7Ag Target at High Levels

A lentiviral overexpression vector expressing MG-7Ag was constructed, as shown in Figure 3(a), and the virus was packaged. After the virus titer was measured, it was transfected into cultured DCs. At 48 h after transfection, total RNA was isolated from DCs, and MG-7Ag expression was evaluated by qPCR.  Figure 3(b) shows that total RNA was isolated from the dendritic cell (DC) vaccine, reverse transcribed to cDNA, and amplified by quantitative polymerase chain reaction to evaluate MG-7Ag expression. The results showed that the expression of MG-7Ag was significantly high in DCs but not in the control group, which indicated that our antigen was successfully expressed in DCs.

### 4.4. Effect of DC Vaccine In Vitro

DCs were pulsed with MG-7Ag and CD3+ T cells were coincubated with MG-7Ag-loaded DCs or unloaded DCs to induce CTL cells. The CTL cells and the target cells KATO-3 and MKN45 were then mixed at a ratio of 10 : 1, 5 : 1, and 1 : 1, respectively, after 16 h, and total CTL cytotoxicity was detected by CCK-8 assay. The results showed that CTLs sensitized by the MG-7Ag DC vaccine had extraordinary cytotoxic effects on both KATO-3 and MKN45 cells. The experimental results at the cellular level showed that the DC vaccine expressing MG-7 had a marked inhibitory effect on the cell line expressing MG-7, as shown in Figure 4.

In lactate dehydrogenase-based cytotoxicity assays, CD3+ T cells stimulated with MG-7 antigen (MG-7Ag)-loaded DCs or unloaded DCs (NC group) were tested against KATO-3, MKN45, and SNU16 cells at various effector-target ratios. Data are expressed as the percentage of specific lysis ±standard deviation (SD) (*n* = 3).

### 4.5. Effect of DC Vaccine In Vivo

To further verify the cytotoxic effect of CTLs sensitized by the DC vaccine, we conducted animal experiments. The MG-7Ag-pulsed DC vaccine or unpulsed DC vaccine was cocultured to induce CTLs. After the mouse PDX model was constructed, the mice in each group were administered CTL saline solution (MG-7Ag-loaded DC vaccine and NC groups) and saline solution (control group) once a day through the tail vein for 3 consecutive days. The mouse tumor volume and mouse bodyweight were then measured every 2 d for 22 d. On day 22, the mouse weight and tumor volume were measured to observe the antitumor effect of CTLs. Compared to the control and NC groups, the DC vaccine loaded with MG-7Ag significantly inhibited the growth of tumors, albeit the weight of the mice was not markedly altered, as shown in Figure 5.

## 5. Conclusions

In this study, we develop a lentiviral vector-programmed DC vaccine with high antitumor responses. By transfecting with a lentiviral vector, the DC vaccine is loaded with MG-7 antigen (MG-7Ag). Three representative gastric cancer cell lines, such as KATO-3, MKN45, and SNU16, are used to estimate the in vitro cytotoxic effect of the MG-7Ag DC vaccine. Furthermore, we examine the in vivo antitumor efficacy of specific cytotoxic T lymphocytes (CTLs) induced by the MG-7Ag DC vaccine in patient-derived xenograft (PDX) mice models. The current data demonstrate that the MG-7Ag DC vaccine induced a potent CTL activity. From the experimental results, it can be observed that those CTLs have a significant cytotoxic effect on both KATO-3 and MKN45 with high level of the MG-7 expression. Also, the MG-7Ag DC vaccine-mediated CTLs significantly inhibit the growth of tumor xenografts in nude mice. We suggest that the MG-7Ag DC vaccine can activate the cytotoxic effect of lymphocytes and can be employed as a vaccine in gastric cancer immunotherapy.

## Figures and Tables

**Figure 1:** Relative level of MG-7Ag.

**Figure 2:** DCs express high levels of surface markers: (a) CD80 FITC-A; (b) CD83 PE-A; (c) CD86 PC5.5-A; (d) HLA-DR APC-A.

**Figure 3:** MG-7Ag DCs express high levels of MG-7Ag target: (a) restriction digestion and electrophoresis results of MG-7 antigen (MG-7Ag) overexpressing lentiviral expression vector; (b) MG-7Ag expression.

**Figure 4:** The inhibitory effect of the dendritic cell (DC) vaccine loaded with MG-7 on gastric cancer cells, KATO-3, MKN45, and SNU16.

**Figure 5:** Changes in the PDX model of gastric cancer on day 22: (a) tumor volume; (b) mouse bodyweight.

## Data Availability

The data used to support the findings of this study are available from the corresponding author upon request.
